# Shikonin suppresses proliferation and induces apoptosis in endometrioid endometrial cancer cells via modulating *miR-106b*/PTEN/AKT/mTOR signaling pathway

This article has been retracted.

**DOI:** 10.1042/BSR20171546

**Published:** 2018-04-13

**Authors:** Caimei Huang, Guohua Hu

**Affiliations:** 1 Department of Traditional Chinese Medicine, Shanghai Changning Maternity and Infant Health Hospital, Shanghai 200051, China; 2 Gynecology of Traditional Chinese Medicine, Shanghai Municipal Hospital of Traditional Chinese Medicine Affiliated to Shanghai TCM University, Shanghai 200071, China

**Keywords:** ant-cancer, endometrioid endometrial cancer, microRNAs, miR-106b/PTEN/AKT/mTOR signaling pathway, Shikonin

## Abstract

Shikonin, a natural naphthoquinone isolated from a traditional Chinese medicinal herb, which exerts anticancer effects in various cancers. However, the molecular mechanisms underlying the therapeutic effects of shikonin against endometrioid endometrial cancer (EEC) have not yet been fully elucidated. Herein, we investigated anticancer effects of shikonin on EEC cells and explored the underlying molecular mechanism. We observed that shikonin inhibits proliferation in human EEC cell lines in a dose-dependent manner. Moreover, shikonin-induced apoptosis was characterized by the up-regulation of the pro-apoptotic proteins cleaved-Caspase-3 and Bax, and the down-regulation of the anti-apoptotic protein Bcl-2. Microarray analyses demonstrated that shikonin induces many miRNAs’ dysregulation, and *miR-106b* was one of the miRNAs being most significantly down-regulated. *miR-106b* was identified to exert procancer effect in various cancers, but in EEC remains unclear. We first confirmed that *miR-106b* is up-regulated in EEC tissues and cells, and knockdown of *miR-106b* suppresses proliferation and promotes apoptosis. Meanwhile, our results validated that the restored expression of *miR-106b* abrogates the antiproliferative and pro-apoptotic effects of shikonin. We also identified that *miR-106b* targets phosphatase and tensin homolog (*PTEN*), a tumor suppressor gene, which in turn modulates AKT/mTOR signaling pathway. Our findings indicated that shikonin inhibits proliferation and promotes apoptosis in human EEC cells by modulating the *miR-106b*/PTEN/AKT/mTOR signaling pathway, suggesting shikonin could act a potential therapeutic agent in the EEC treatment.

## Introduction

Endometrial cancer (EC) is the most common gynecologic malignancy in the developed countries [1]. Statistical analysis has shown that approximately 142000 women suffered from EC globally every year, and approximately 42000 women die from this disease [2]. Amongst these EC cases, approximately 80% are endometrioid EC (EEC) [3], which is mainly treated with combination of surgery and adjuvant chemotherapy, radiotherapy or hormone therapy. However, these conventional chemotherapy and radiotherapy cause side effects for advanced patients or yield suboptimal results for those with recurrent EEC [4]. Therefore, it is a strong medical need to develop a novel therapeutic agent against EEC that exhibit reduced toxicity and increased efficiency.

Shikonin, an active naphthoquinone of Zi Cao, derived from the roots of the herb *Lithospermu erythrorhizon* that has been used in traditional Chinese medicine to treat skin diseases, burns and sore throats due to its antimicrobial and anti-inflammatory activities [5,6]. Recently, it has been identified that shikonin exerts various anticancer effects such as inhibiting proliferation and promoting apoptosis in human lung adenocarcinoma cells, suppressing prostate cancer cell metastasis, weakening migration and invasion in human breast cancer cells [7–10]. Liu et al. [11] uncovered that shikonin protects against concanavalin A-induced acute liver injury via inhibition of the JNK pathway in mice. Jang et al. [8] demonstrated that shikonin attenuates human breast cancer cells migration and invasion via suppressing matrix metalloproteinase-9 activation. Wang et al. [12] clarified that shikonin inhibits interleukin-1β-induced chondrocytes’ apoptosis through modulating PI3K/AKT signaling pathway. Furthermore, it has been reported that shikonin possesses the suppressive effects on EEC cells via promoting apoptosis and blocking cell cycle [13]. However, the molecular mechanism of the anticancer effects of shikonin on EEC cells remain unclear.

miRNAs are a group of endogenous, non-coding small RNAs of 22–25 nts, which serve as a regulator of gene expression at the post-transcriptional level via suppressing translation or promoting RNA degradation. There is a growing body of evidence that miRNAs are involved in a variety of biological and pathological processes including cellular differentiation, proliferation, apoptosis, and carcinogenesis [14–16]. In recent years, it has been extensively reported that some Chinese medicinal herbs exert antitumor effects in different cancers via regulating miRNA expression profiles [17,18]. Curcumin suppresses cell growth, invasion, tumor growth in colorectal cancer and *in vivo* metastasis by regulation of *miR-21* [19]. Zhang et al. [20] illustrated that honokiol inhibits bladder tumor growth by blocking the EZH2/*miR-143* axis. In addition, shikonin has been identified to act as a potential therapeutic agent to treat human glioblastoma through regulating miRNA expression profiles [21]. Against this background, we hypothesized that shikonin exerts anticancer effect on human EEC via modulating miRNA expression.

In the present study, we investigated the anticancer effects of shikonin on EEC cells and explored the underlying molecular mechanism by identifying shikonin-induced miRNA dysregulations. Our results suggested that shikonin may possess anticancer effects on EEC via mediating *miR-106b*/phosphatase and tensin homolog (PTEN)/AKT/mTOR signaling pathway and act as a potential therapeutic agent for the treatment of EEC.

## Materials and methods

### Patient tissue specimens

Twenty EEC tissues and twenty normal endometrial samples were collected from patients who underwent surgical resection at Gynecology of Traditional Chinese Medicine, Shanghai Municipal Hospital of Traditional Chinese Medicine Affiliated to Shanghai TCM University (Shanghai, China) between April 2016 and April 2017. None of the patients had received pre-operative radiotherapy or chemotherapy prior to surgical resection. The tumor specimens were independently confirmed by two pathologists. Fresh specimens were snap-frozen in liquid nitrogen and stored at −80°C immediately after resection for subsequent RNA extraction. The project protocol was approved by the Ethics Committee of Shanghai TCM University. All patients provided written informed consents for the use of the tumor tissues for clinical research.

### Cell culture and treatment

The human EEC cell lines Ishikawa, HEC-1A, KLE, and RL95-2 were obtained from American Type Culture Collection (ATCC, Manassas, VA, U.S.A.) and one normal endometrial cell (ESC) were obtained from the Tumor Cell Bank of the Chinese Academy of Medical Science (Peking, China), and maintained in DMEM, supplemented with streptomycin (100 IU/ml), penicillin (100 IU/ml, Sigma, St. Louis, MO), 2 mM glutamine, and 10% FBS (Gibco BRL, Grand Island, NY). Cells (1 × 10^4^/well) were seeded in 96-well plates for 24 h and then incubated with shikonin (10–20 μM) at 24 h for further measurements. Shikonin was purchased from National Institute for the Control of Pharmaceutical and Biological Products (Beijing, China) with purity >99%. Shikonin was dissolved in DMSO (Sigma) and stored at −20°C.

### Cell viability analysis

The Cell Counting Kit-8 (CCK-8) assay was used to measure proliferation of cells according to the manufacturer’s instruction (Beyotime Institute of Biotechnology, Shanghai, China). The cells (5 × 10^4^ cells/well) were seeded in 96-well plate with 100 μl DMEM medium supplemented with 10% FBS. After 48 h incubation, 10 μl CCK-8 reagent dissolved with 100 µl DMEM was added to each well and continuously cultured for 1 h in 5% CO_2_ (Thermo). The absorbance rate at 450 nm were measured by Microplate Reader (Bio–Rad, U.S.A.). All experiments were performed in quintuplicate on three separate occasions.

### Apoptosis analysis

The flow cytometry analysis was used to measure cell apoptosis. The cells were treated with shikonin for 24 h, and were then collected and washed twice with PBS. After treatment with trypsin, cells were fixed with 70% ice-cold methanol at 4°C for 30 min. Cells were resuspended in binding buffer and stained with 5 μl of AnnexinV-FITC (BD, Mountain View, CA, U.S.A.) and 1 μl of propidium iodide (PI, 50 μg/ml) (BD, Mountain View, CA, U.S.A.). Flow cytometric evaluation was performed within 5 min. Stained cells were analyzed using flow cytometry (BD, FACSCalibur, CA, U.S.A.). The measurements were performed independently for at least three times with similar results.

### miRNA microarray analysis

miRNA microarray analysis was used to evaluate miRNA expression in cells after treatment with shikonin. Total RNA was isolated from cells using TRIzol reagent (Molecular Research Center, Inc., Cincinnati, OH, U.S.A.) and purified by RNeasy MinEluted Cleanup kit (QIAGEN, Germany) according to manufacturer’s instructions. After measuring the quantity of RNA using a NanoDrop 1000 (Youpu Scientific Instrument Co., Ltd., Shanghai, China), the samples were labeled using the miRCURY™Hy3™/Hy5™ Power labeling kit (Exiqon, Vedbaek, Denmark) and hybridized on a miRCURY™ LNA Array (version 18.0, Exiqon, Vedbaek, Denmark). After washing, the slides were scanned using an Axon GenePix 4000B microarray scanner (Axon Instruments, Foster City, CA, U.S.A.). Scanned images were then imported into the GenePix Pro6.0 program (Axon Instruments) for grid alignment and data extraction. Replicated miRNAs were averaged, and miRNAs with intensities ≥50 in all samples were used to calculate a normalization factor. Expressed data were normalized by median normalization. After normalization, the miRNAs that were significantly differentially expressed were identified by Volcano Plot filtering. Hierarchical clustering was used to determine the differences in the miRNA expression profiles amongst different genes and samples using MEV software (version 4.6; TIGR, Microarray Software Suite4, Boston, U.S.A.).

### RNA extraction and real-time quantitative PCR

Total RNA was extracted from culture cells using TRIzol Reagent (Invitrogen) and quantitated with UV spectrophotometer (SmartSpec plus). The High Capacity cDNA Synthesis Kit (Applied Biosystems) was used to synthesize cDNA with miRNA-specific primers. The primers for *miR-106b* and the internal control *RNU44* gene were obtained from Ambion. The real-time quantitative PCR (RT-qPCR) was carried out using TaqMan Gene Expression Assay (Applied Biosystems) on an Applied Biosystems 7500 Real-Time PCR machine. The 2^−ΔΔ*C*^_t_ method was used to determine the miRNAs relative expression. All reactions were performed in triplicate.

### Western blot analysis

The cells were lysed as described previously [22]. The protein concentration was measured using BCA protein assay kit (Pierce, Rockford, IL). Total proteins (60 μg) were separated in SDS/polyacrylamide gels (10% gels) (Sigma–Aldrich, St. Louis, MO) and then transferred on to PVDF membranes (BD Pharmingen, San Diego, CA). After blocking with 5% non-fat milk at room temperature for 1 h, the PVDF membranes were incubated primary antibodies against cleaved-Caspase-3, Bax, Bcl-2, PTEN, p-AKT, AKT, p-mTOR, and mTOR at 4°C overnight. These antibodies were obtained from Santa Cruz Biotechnology (Santa Cruz, CA, U.S.A.). β-actin (Sigma, St. Louis, MO, U.S.A.) was used as an internal control. Horseradish peroxidase-conjugated (HRP) antibodies (Santa Cruz Biotechnology, Santa Cruz, CA) were used as the secondary antibodies. Subsequently, the protein bands were scanned on the X-ray film using the ECL detection system (PerkinElmer Life and Analytical Sciences, Boston, MA). The alpha Imager software (Alpha Innotech Corporation, San Leandro, CA) was used to measure relative intensity of each band on Western blots. The measurements were performed independently for at least three times with similar results.

### Luciferase reporter assay

The potential binding site between PTEN and *miR-106b* was identified using TargetScan (http://www.targetscan.org). The *miR-106b* mimics/inhibitor and corresponding negative control (NC) were synthesized by RiboBio (Guangzhou, China). The wild-type (wt) PTEN-3′-UTR and mutant (mut) PTEN-3′-UTR containing the putative binding site of *miR-106b* were established (Figure 5A) and cloned in the firefly luciferase expressing vector pMIR-REPORT (Ambion, U.S.A.). Site-directed mutagenesis of the PTEN 3′-UTR at the putative *miR-106b* binding site was performed by a QuikChange Kit (Qiagen). For the luciferase assay, Ishikawa cells at a density of 2 × 10^5^ per well were seeded into 24-well plates and co-transfected with 0.8 μg of pMIR-PTEN-3′-UTR or pMIR-PTEN-mut-3′-UTR, 50 nM *miR-106b* mimic/inhibitor or corresponding mimic NC using Lipofectamine 2000 reagent (Invitrogen). The relative firefly luciferase activity normalized with *Renilla* luciferase was measured 48 h after transfection by using the Dual-Light luminescent reporter gene assay (Applied Biosystems).

### Statistical analysis

All statistical analyses were performed using SPSS 14.0 software (Chicago, IL). Each experiment was repeated at least three times. Numerical data are presented as the mean ± S.E.M. The comparison between data was calculated using Student’s *t*test (between two groups) and one-way ANOVA and Tukey’s multiple comparison tests (between multiple groups). *P*-value of <0.05 was considered significant and <0.01 was considered very significant.

## Results

### Shikonin inhibits the growth of human EEC cells

To explore the antiproliferative effect of shikonin on EEC cells, the human EEC cell lines Ishikawa, HEC-1A, KLE, and RL95-2 were treated with various concentrations of shikonin (0, 1, 2, 4, 8, 10, and 20 μM) for 24 h and the cell viability was evaluated by CCK-8 assay. As shown in Figure 1A–D, shikonin markedly reduced cell viability in a dose-dependent manner compared with blank group in all human EEC cell lines (*P*<0.01). The shikonin IC_50_ values (the concentration of 50% inhibition cell viability) were 3.63, 4.81, 8.22, and 8.96 μM in Ishikawa, HEC-1A, KLE, and RL95-2, respectively. The most sensitive EEC cell lines Ishikawa and HEC-1A for shikonin were selected in the subsequent experiments. To determine the induction of cell apoptosis by shikonin in the human EEC cell lines, the Ishikawa and HEC-1A cells treated with 5 μM of shikonin for 24 h, and the apoptotic cells were evaluated using flow cytometric analysis. Compared with blank group, shikonin treatment significantly increased apoptotic cells in both Ishikawa and HEC-1A cells (*P*<0.01; Figure 1E). To further explore the molecular mechanisms of shikonin-induced apoptosis, we performed the Western blot analysis to measure the expression levels of the apoptosis-related proteins in Ishikawa and HEC-1A cells treated with 5 μM of shikonin for 24 h. We found that shikonin markedly up-regulated the pro-apoptotic proteins (cleaved-Caspase-3 and Bax) and down-regulated the anti-apoptotic protein (Bcl-2) compared with blank group (*P*<0.01; Figure 1F,G). Collectively, we first demonstrated that shikonin inhibits proliferation and induces apoptosis in human EEC cells.

**Figure 1:** The suppressive effects of shikonin on human EEC cells (**A**–**D**) The human EEC cell lines Ishikawa, HEC-1A, KLE, and RL95-2 were treated with various concentrations of shikonin (0, 1, 2, 4, 8, 10, and 20 μM) for 24 h and the cell viability was measured by the CCK-8 assay. (**E**) The flow cytometric analysis was used to determine the apoptotic cells in both Ishikawa and HEC-1A cells after treatment with 5 μM of shikonin for 24 h. (**F**,**G**) The Ishikawa and HEC-1A cells treated with 5 μM of shikonin for 24 h, the Western blot analysis to detect the expression levels of the apoptosis-related proteins (cleaved-Caspase-3, Bax, and Bcl-2). β-actin was used as an internal control for protein loading. Data are represented as means ± S.D. of three independent experiments (*P<0.05, **P<0.01 compared with blank group).

### Shikonin induces the aberrant expression of miRNAs in human EEC cells

Recently, many Chinese medicinal herbs were demonstrated to harbor the antitumor effects in various cancers through modulating miRNA expression profiles [17,18]. To investigate whether shikonin suppresses EEC cells’ growth via regulating miRNAs expression, we performed microarray analysis to determine miRNA levels in EEC cells after treatment with shikonin (5 μM) for 24 h. As shown in Figure 2A, compared with blank group, shikonin treatment resulted in aberrant expression of miRNAs, and *miR-106b* is one of the miRNAs being most significantly down-regulated in EEC cells. It is well reported that *miR-106b* has been identified to act as an oncogene in various cancers including breast cancer, osteosarcoma, and hepatocellular carcinoma [23–25]. To explore the role of *miR-106b* in the suppressive effects of shikonin on EEC cells, the Ishikawa cells were treated with various concentration of shikonin (0, 1, 2, 5, and 10 μM) for 24 h and *miR-106b* levels were quantitated by qRT-PCR. We observed that shikonin reduced the *miR-106b* expression in a dose-dependent manner in Ishikawa cells (Figure 2B). These data suggested that shikonin may exert anticancer effects via suppressing the expression of oncogenic *miR-106b* in EEC cells.

**Figure 2:** Shikonin induces the aberrant expression of miRNAs in human EEC cells (**A**) The EEC cells were treated with shikonin (5 μM) for 24 h, and then microarray analysis was conducted to identify miRNA expression profiles. The color code is linear within the heat map: blue represents the lowest level of expression and red the highest. (**B**) The qRT-PCR analysis was performed to determine the *miR-106b* expression in Ishikawa cells treated with different concentration of shikonin (0, 1, 2, 5, and 10 μM) for 24 h (*P<0.05, **P<0.01 compared with blank group). (**C**) *miR-106b* was identified by qRT-PCR analysis in EEC tissues (*n*=20) and normal endometrial samples (*n*=20) (**P<0.01 compared with normal endometrial samples). (**D**) The qRT-PCR analysis was used to detect *miR-106b* level in EEC cell lines Ishikawa, HEC-1A, KLE, RL95-2, and one normal endometrial cell (ESC) (**P<0.01 compared with ESC). Data are represented as means ± S.D. of three independent experiments.

### Knockdown of *miR-106b* inhibits EEC cells apoptosis

*miR-106b* has been demonstrated to function as an oncogene in many cancers [23–25], but its role in EEC has yet to be elucidated. To investigate the role of *miR-106b* in EEC, we performed the qRT-PCR to determine *miR-106b* expression in EEC tissues and found that *miR-106b* is dramatically up-regulated in cancer tissues compared with normal tissues (*P*<0.01; Figure 2C). Moreover, our results further verified that *miR-106b* is also significantly overexpressed in EEC cell lines (Ishikawa, HEC-1A, KLE, and RL95-2) compared with ESC cell (*P*<0.01; Figure 2D). These results indicated that *miR-106b* may play an oncogenic role in the development of EEC. To further explore the effects of *miR-106b* on EEC cells, the Ishikawa and HEC-1A cells were transfected with *miR-106b* inhibitor or inhibitor NC, and then cell viability and apoptotic cells were measured by CCK-8 assay and cytometric analysis, respectively. As shown in Figure 3A–C, compared with inhibitor NC, knockdown of *miR-106b* markedly reduces cell viability and increases apoptotic cells (*P*<0.01). In addition, our results demonstrated that knockdown of *miR-106b* up-regulated the pro-apoptotic proteins (cleaved-Caspase-3 and Bax) and down-regulated the anti-apoptotic protein (Bcl-2) compared with inhibitor NC group (Figure 3D,E). Taken together, these findings suggested that *miR-106b* is overexpressed in EEC tissues and cells, and function as an oncogene in EEC.

**Figure 3:** Knockdown of *miR-106b* suppresses EEC cells apoptosis (**A**,**B**) The Ishikawa or HEC-1A cells were transfected with *miR-106b* inhibitor or inhibitor NC, and cell viability was measured using CCK-8 post treatment at 1, 2, 3 and 4 days, respectively. (**C**) The cytometric analysis used to measure apoptotic cells in Ishikawa and HEC-1A cells treated with *miR-106b* inhibitor or inhibitor NC. (**D**,**E**) After transfection with *miR-106b* inhibitor or inhibitor NC, the Western blot analysis was used to detect the expression levels of the apoptosis-related proteins (cleaved-Caspase-3, Bax, and Bcl-2). β-actin was used as an internal control for protein loading (**P<0.01 compared with inhibitor NC). Data are represented as means ± S.D. of three independent experiments.

### Overexpression of *miR-106b* attenuates the suppressive effects of shikonin

Based on the above results, our data demonstrated that *miR-106b* was down-regulated in Ishikawa cells after treatment with shikonin. Moreover, *miR-106b* was identified to act as an oncogene in EEC. Therefore, we speculated whether shikonin possesses the antiproliferation effects on EEC cells through modulating *miR-106b* expression. Then, the Ishikawa or HEC-1A cells were transfected with *miR-106b* mimics or mimics NC, and treated with shikonin (5 μM) for 24, 48, and 72 h. Subsequently, the cellular proliferation and apoptotic cells were measured by CCK-8 assay and cytometric analysis, respectively. We found that shikonin treatment dramatically inhibits cell proliferation and promotes apoptosis in shikonin + mimic NC group compared with blank group, but these suppressive effects of shikonin on EEC cells were abolished by overexpression of *miR-106b* in shikonin + *miR-106b* mimic group (*P*<0.01; Figure 4A–D). These results indicated that the shikonin may exert suppressive effects on EEC cells via regulating *miR-106b* expression. However, the precise molecular mechanisms by which shikonin represses EEC cell growth needs further research.

**Figure 4:** Overexpression of *miR-106b* attenuates the suppressive effects of shikonin (**A** and **C**) The Ishikawa or HEC-1A cells were transfected with *miR-106b* mimics or NC, and then treated with shikonin (5 μM) for 24, 48, and 72 h; the CCK-8 was assay used to measure cellular proliferation, respectively. (**B** and **D**) After transfection with *miR-106b* mimics or NC, the apoptotic cells were measured by cytometric analysis in Ishikawa or HEC-1A cells treated with shikonin (5 μM) for 24 h. Data are represented as means ± S.D. of three independent experiments (*P<0.05, **P<0.01 compared with blank group, ^##^*P*<0.01 compared with shikonin + mimics NC group).

### *miR-106b* inhibits PTEN expression by directly targetting its 3′-UTR

Previous studies uncovered that *miR-106b* could post-transcriptionally inhibit PTEN expression in different cancer cells, such as pituitary adenoma, breast cancer, and colorectal cancer [23,26–28], but whether PTEN was a direct target of *miR-106b* in human EEC cells remains to be further elucidated. Moreover, we further predicted the target genes of *miR-106b* using TargetScan, and identified PTEN as a potential target of *miR-106b* (Figure 5A). Subsequently, we constructed luciferase-reporter plasmids that contain the wt or mut 3′-UTR segments of PTEN (Figure 5A). The wt or mut reporter plasmid was co-transfected into Ishikawa cells along with *miR-106b* mimics/inhibitor or NC, and measured the luciferase activity. We observed that *miR-106b* mimic dramatically suppressed the luciferase activity compared with the mimic NC, but *miR-106b* inhibitor significantly increased the luciferase activity compared with the inhibitor NC (*P*<0.01; Figure 5D). Additionally, *miR-106b* did not inhibit the luciferase activity of the reporter vector containing 3′-UTR of PTEN with mutations in the miR-106b-binding site (Figure 5D). To further validate that the PTEN level is regulated by *miR-106b*, the Ishikawa or HEC-1A cells were transfected with *miR-106b* mimic/inhibitor or NC and Western blot was used to detect PTEN level. As shown in Figure 5B,C, up-regulation of *miR-106b* reduced the PTEN protein level compared with NC, conversely, knockdown of *miR-106b* increased the PTEN protein expression. These data indicated that *miR-106b* suppresses PTEN expression by directly targetting its 3′-UTR in human EEC cells.

**Figure 5:** PTEN is a target of *miR-106b* in EEC cells (**A**) The PTEN 3′-UTR region containing the wt or mut binding site for *miR-106b*. (**B**,**C**) The Ishikawa or HEC-1A cells transfected with the *miR-106b* mimic/inhibitor or corresponding NC, and the PTEN expression was measured by Western blot analysis. β-actin was used as an internal control for protein loading. (**D**) The relative luciferase activity of PTEN wt or mut 3′-UTR in Ishikawa cells after transfection with the *miR-106b* mimic/inhibitor or corresponding NC. Data are represented as means ± S.D. of three independent experiments (**P<0.01 compared with mimics NC, ^##^*P*<0.01 compared with inhibitor NC).

### Overexpression of PTEN inhibits human EEC cell growth

To investigate the role of PTEN in human EEC cells, the Ishikawa or HEC-1A cells were transfected with pc-DNA-PTEN or pc-DNA-vector and then cell viability and apoptosis were measured by CCK-8 assay and flow cytometric analysis, respectively. As shown in Figure 6A, the PTEN protein expression was obviously u-pregulated in both Ishikawa and HEC-1A cells transfected with pc-DNA-PTEN compared with pc-DNA-vector (*P*<0.01). Moreover, our results showed that overexpression of PTEN significantly suppressed proliferation and promotes apoptosis in both Ishikawa and HEC-1A cells compared with pc-DNA-vector (*P*<0.01; Figure 6B,C). These results indicated that PTEN may act as a tumor suppressor gene in human EEC cells.

**Figure 6:** Overexpression of PTEN inhibits human EEC cell growth The Ishikawa or HEC-1A cells were transfected with pc-DNA-PTEN or pc-DNA-vector. (**A**) The PTEN protein expression was measured by Western blot analysis. (**B**,**C**) The CCK-8 assay and flow cytometric analysis were used to evaluate the cell viability and apoptosis in Ishikawa and HEC-1A cells, respectively. Data are represented as means ± S.D. of three independent experiments (**P<0.01 compared with blank, ^##^*P*<0.01 compared with pc-DNA-vector).

### Shikonin suppresses the PTEN/AKT/mTOR signaling pathway via down-regulation of *miR-106b*

AKT/mTOR signaling which is negatively modulated by PTEN is a key pathway in cell survival, cellular proliferation, and tumor growth [29–31]. Recent studies demonstrated that *miR-106b* promotes the cell proliferation, invasion, and migration in a variety of cancers via modulating PTEN/PI3K/AKT signaling pathway [23,26,27]. Inspired by these studies, we hypothesized whether shikonin-induced *miR-106b* down-regulation modulates PTEN/AKT/mTOR signaling pathway in EEC cells. To verify this hypothesis, after transfection with or without *miR-106b* mimics, the Ishikawa or HEC-1A cells were treated with shikonin (5 μM) for 24 h and PTEN, AKT and mTOR were identified using Western blot. Our results showed that shikonin treatment markedly increased PTEN expression and decreased the p-AKT and p-mTOR levels compared with blank group in both Ishikawa and HEC-1A cells, but this shikonin-blocked PTEN/AKT/mTOR pathway was reactivated by overexpression of *miR-106b* (*P*<0.01; Figure 7A–D). These data illustrated that shikonin is able to repress the PTEN/AKT/mTOR signaling pathway in human EEC cells, but it could be reactivated by *miR-106b* overexpression. Taken together, these results suggested that shikonin blocks PTEN/AKT/mTOR signaling pathway via suppressing *miR-106b* expression in human EEC cells.

**Figure 7:** Shikonin blocks the PTEN/AKT/mTOR signaling pathway via suppressing *miR-106b* (**A** and **C**) After transfection with or without *miR-106b* mimic, the Ishikawa or HEC-1A cells were treated with shikonin (5 μM) for 24 h, and then the expression levels of PTEN, AKT, p-AKT, mTOR, and p-mTOR were measured using Western blot analysis. (**B** and **D**) Quantitation of PTEN, AKT, p-AKT, mTOR, and p-mTOR ratios relative to controls in Ishikawa or HEC-1A cells, respectively. Data are represented as means ± S.D. of three independent experiments (**P<0.01 compared with blank, ^##^*P*<0.01 compared with shikonin).

## Discussion

Emerging evidence revealed that shikonin exerts the anticancer effect in various cancers [7–11]. However, whether shikonin exhibits such anticancer functions when used in the context of the treatment of human EEC remains unclear. In the present study, we investigated the suppressive effects of shikonin on EEC cells, and explored the underlying molecular mechanisms. We observed that shikonin suppresses proliferation of EEC cells in a dose-dependent manner, and induced apoptosis via regulation of apoptosis-related proteins. Microarray analyses uncovered that shikonin induces a large set of miRNAs dysregulation, and the *miR-106b* was one of the miRNAs being most significantly down-regulated. Moreover, we confirmed that *miR-106b* is up-regulated in EEC tissues and cells, and the suppressive effects of shikonin were abrogated by overexpression of *miR-106b* in EEC cells. More importantly, our results indicated that shikonin represses proliferation and induces apoptosis in ECC cells via modulating *miR-106b*/PTEN/AKT/mTOR axis.

The naturally derived products with anticancer effects have been widely utilized as the source of many medically beneficial drugs, such as curcumin, camptothecin, luteolin, honokiol, isoflavone, matrine, xanthoangelol, and shikonin [7,32,33]. Xanthoangelol, isolated from *Angelica keiskei* roots, which suppressed tumor growth, metastasis to the liver and lung, and tumor-associated macrophage expression in tumors [33]. Icaritin, a traditional Chinese herbal medicine, which induces sustained ERK1/2 activation, represses human EC cells growth and promotes apoptosis [34]. With regard to shikonin, it has been identified to act as a potential anticancer agent against various cancers, including human lung adenocarcinoma, prostate cancer, and breast cancer [7–10]. However, the anticancer effects of shikonin on EEC were rarely reported. In the present study, our results showed that shikonin inhibits EEC cell growth in a dose-dependent manner, and induces apoptosis in EEC cells via activating the intracellular apoptotic signaling pathway. These data indicated that shikonin exerts the antiproliferative property in EEC cells and could be developed as a potential therapeutic agent against human EEC.

Growing evidence demonstrated that many miRNAs play key role in a variety of cancers, while the anticancer effects of traditional Chinese herbal medicine that operate through targetting miRNAs have also been widely reported. Zeng et al. [35] revealed that camptothecin induces human cervical cancer cells’ and human prostate cancer cells’ apoptosis via *miR-125b*-mediated mitochondrial pathways. Liu et al. confirmed that berberine could target the *miR-21*/PDCD4 axis, and improves cisplatin sensitivity in ovarian cancer cells [17]. In addition, shikonin has been demonstrated to act as a therapeutic agent to treat human glioblastoma via regulating miRNAs expression profiles [21]. In the present study, we performed microarray analysis to identify miRNAs expression in EEC cells treated with shikonin, and found that shikonin alters a large set of miRNAs and *miR-106b* was one of the miRNAs being most significantly down-regulated. Previous studies have demonstrated that *miR-106b* function as an oncogene in different cancers, such as breast cancer, osteosarcoma, and hepatocellular carcinoma [23–25]. Therefore, the *miR-106b* attracts us to investigate its role in EEC cells. Our results first demonstrated that *miR-106b* functions as an oncogene in EEC, and knockdown of *miR-106b* suppresses cell proliferation and apoptosis via modulating the intracellular apoptotic signaling pathway. Against this background, we hypothesized that shikonin may exert the anticancer effect in EEC through suppressing this oncogenic miRNA. Our results confirmed that the antiproliferative and pro-apoptotic effects of shikonin on EEC cell were abolished by *miR-106b* overexpression. These data suggested that shikonin may exert the suppressive effects on EEC cells via down-regulating *miR-106b*. However, the precise molecular mechanism needs further research to be understood deeply.

AKT/mTOR signaling plays a central role in cell survival, cellular proliferation, and tumor growth [29–31], which was negatively regulated by PTEN [36,37]. Previous studies identified that *miR-106b* inhibits PTEN expression through directly targetting its 3′-UTR in many cancer cells [23,26,27]. In the present study, our results also verified that PTEN is a target of *miR-106b* in ECC cells. In addition, overexpression of PTEN also inhibits proliferation and induces apoptosis in both Ishikawa and HEC-1A cells. It is well reported that *miR-106b* promotes the cell proliferation, invasion, and migration via regulating PTEN/PI3K/AKT signaling pathway in various cancers [23,26,27]. Then, we speculated that shikonin may exert suppressive effects on EEC cells via modulating PTEN/AKT/mTOR signaling pathway by suppressing *miR-106b* expression. As expected, shikonin treatment could inhibit the PTEN/AKT/mTOR signaling pathway in human EEC cells, but it was reactivated by *miR-106b* up-regulation. Collectively, these data indicated that shikonin blocks PTEN/AKT/mTOR signaling pathway via inhibiting *miR-106b* expression in human EEC cells (Figure 8).

**Figure 8:** The schematic mechanism The schematic diagram illustrates that shikonin treatment induces the down-regulation of *miR-106b* in EEC cells, and then results in the up-regualtion of PTEN. Subsequently, up-regualtion of PTEN can antagonize PI3K signal transduction by dephosphorylating the PI3K phosphorylation products (PI3,4,P_2_ and PI3,4,5,P_3_), leading to the down-regulation of AKT/mTOR, and regulate cell survival and apoptosis.

In conclusion, our results demonstrated that shikonin inhibits cell growth in EEC cells via regulating the intracellular apoptotic signaling pathway. Additionally, we first demonstrated that *miR-106b* acts as an oncogene by targetting the tumor suppressor gene *PTEN* in EEC cells. More importantly, our results uncovered that shikonin possessed the suppressive effects on ECC cells via blocking *miR-106b*/PTEN/AKT/mTOR signaling pathway, suggesting shikonin could act as a promising anticancer agent for EEC treatment.

## Abbreviations

CCK-8: cell counting kit-8
DMEM: Dulbecco’s Modified Eagle’s Medium
EEC: endometrioid endometrial cancer
mut: mutant
NC: negative control
PTEN: phosphatase and tensin homolog
wt: wild-type
